The article "Effects of Psychological Well-Being and Depression on Menopausal Symptoms in Middle-Aged South Korean Women and the Necessity of Exercise" was retracted in 2023. Reasons: signs of a paper mill; suspected computer-generated content; unreliable results or conclusions; lack of ethics approval or compliance.

# Effects of Psychological Well-Being and Depression on Menopausal Symptoms in Middle-Aged South Korean Women and the Necessity of Exercise

**DOI:** 10.1155/2022/6529393

**Published:** 2022-08-08

**Authors:** Sungsim Lee, Sookyoung Jeong, Youngsoon Choi

**Affiliations:** ^1^Department of Nursing, Gangneung Yeongdong College, 357 Gongje-ro, Gangneung-si, Gangwon-do, Republic of Korea; ^2^Department of Nursing, Saekyung College, 197 Hasong-ro, Yeongwol-eup, Yeongwol-gun, Gangwon-do, Republic of Korea; ^3^Department of Nursing, Kangwon National University, 346 Hwangjo-gil, Dogye-eup Samcheck-si, Gangwon-do 25949, Republic of Korea

## Abstract

The purpose of this study was to provide basic data on the health by examining the effects of psychological well-being and depression on menopausal symptoms and the necessity of exercise in middle-aged women. This study is a cross-sectional study using a structured questionnaire. The respondent's consent was obtained prior to data collection, and the investigation period runs from November 1, 2021 to November 30, 2021. The final analysis included 150 as respondents to the study. The tool developed by Yang was used for psychological well-being, the Korean integrated CES-D tool was used for depression, and the Menopause Symptom Index was used for menopausal symptoms. The differences and levels of psychological well-being, depression, and menopausal symptoms according to demographic and sociological characteristics were analyzed using descriptive statistics, *t*-test, and ANOVA. The correlation between psychological well-being, depression, and menopausal symptoms was analyzed by Pearson's correlation, and the effect on menopausal symptoms was analyzed by multiple regression. Because of this study, significant results were found in marital status, religion, economic level, regular exercise, hobbies, personality, and subjective health in the difference in psychological well-being according to general characteristics. In depression, significant results were found in marital status, education level, monthly income, living status, regular exercise, hobbies, stress, personality, and subjective health status. Moreover, age, frequent exercise, hobby, and subjective health all had a significant impact on menopausal symptoms. According to the findings of the regression analysis, the factors influencing menopausal symptoms were, in that order, depression and psychological well-being. Among the factors that showed significant results for menopausal symptoms, exercise is recommended as a factor that can alleviate menopausal symptoms due to individual lifestyle changes, so it is expected to contribute to reducing menopausal symptoms and improving quality of life.

## 1. Introduction

In Korea, the average life expectancy is significantly increasing with the development of medical technology, improvement in living standards, and economic growth [1]. Males in Korea have a life expectancy of 80.5 years, while women have an expectation of 86.5 years, implying that women would live nearly 6 years longer than men [1].

Middle age is a natural event that can be considered a turning point in the life of a woman's typical life cycle. In addition, in modern times, this period is regarded as the second birth to reflect on the meaning of one's health and quality of life [2]. Middle age is a stage of a woman's normal life cycle, and she experiences physiological changes due to aging, including menopause. It is also a turning point in life that requires psychological adaptation in many ways, such as changing roles in the family and coping with conflicts caused by children's studies, work, and marriage [3]. This period is characterized by the most stable and satisfactory period due to the family, social status, and economic leisure that one has achieved. However, it is time to take responsibility for children and elderly parents, as well as for the state and society, to experience diverse and individual symptoms of menopause, such as aging, and to adjust to physical fitness accordingly [2].

Menopause is the transition from genital to nongenital in the process of gradual aging of body tissues. The age varies slightly in each document, but generally refers to 40–60 years. This period refers to the time between the period of endocrine disruption, when menstrual phenomena for reproductive functions such as ovulation and menstruation undergo irregular periods of change, along with the decreased secretion of ovarian hormones, and the period of menopause, when they regain stability [4]. Middle age is a transitional period to old age, during which physical fertility is reduced, and menopause is experienced. It is also a time when various menopausal symptoms such as hot flashes, memory loss, and changes in the genitourinary system are experienced, and the possibility of chronic diseases such as cerebro-cardiovascular disease, joint pain, osteoporosis, and cancer in women increases [5]. Menopausal symptoms due to the decrease of female hormones and factors such as physical, mental, psychological, and sexual are combined, and menopausal symptoms appear in various forms [6]. Menopausal symptoms vary widely over time and across individuals and are perceived positively or negatively [7].

Menopausal symptoms are experienced by 38 to 39% of middle-aged Korean women [8]. Middle-aged women experienced menopausal symptoms in the following order: joint pain, psychoneurotic symptoms, skeletal symptoms, vasomotor symptoms, urogenital symptoms, and cardiovascular symptoms [9]. The main symptoms of menopause are hot flashes, sweating, headache, low back pain, aching limbs, joint pain, nervousness, forgetfulness, incontinence, genital dryness, fatigue, and depression [9]. Menopausal symptoms affect the lives of middle-aged women in various ways. Interruption of menstruation, physical aging, and loss of role experienced by menopausal women make them fall into depression, and these depressive symptoms lose the meaning of life. Depending on how the menopausal symptoms are managed, they may transition to unhealthy health, causing serious diseases or lowering the quality of life [10].

Previous studies on climacteric symptoms of middle-aged women were conducted during the research period using art therapy, fragrance inhalation therapy, religious orientation, quality of life, and self-esteem as variables [11]. However, research on variables for psychological well-being or depression is insufficient. Furthermore, the interpretation of postmortem depression results may vary since prior research that evaluated menopausal symptoms and depression in middle-aged women used a similar experimental study and non-equivalence control post-design [11]. This study investigated the effects of psychological well-being and depression on menopausal symptoms and exercise needs in a descriptive way.

The purpose of this study was to provide basic data on the health by examining the effects of psychological well-being and depression on menopausal symptoms and the necessity of exercise in middle-aged women. The specific objectives are as follows: First, the characteristics of the subject, a sense of psychological fulfillment, and the degree of depression and climacteric symptoms are identified. Second, the degree of psychological well-being and depression according to the characteristics of the subject is identified. Third, the relationship between psychological well-being, depression, and menopausal symptoms of the subject is investigated. Fourth, the effect of psychological well-being and depression on menopausal symptoms is investigated.

## 2. Literature Review

Psychological well-being is a positive cognitive and emotional state in which various factors are integrated. It is a phenomenon of hedonistic pleasure or emotional improvement, which is one of the emotional responses that people who participate in active physical activity report repeatedly after exercise [12, 13]. Despite the fact that this is the basic attitude to have in order to live a normal life, middle-aged women in current times have a low sense of psychological well-being [14]. Kang Hyeon-ju investigated and reviewed life stress and psychological well-being of middle-aged women [15]. Through this, she said, it is necessary to find a way to improve the quality of life by presenting basic data that can promote not only stress but also psychological well-being as they enter middle age. Song et al. [16] proposed that middle-aged women should develop their psychological well-being in order to experience ultimate human happiness through rhythmic movements at a time when they may be afflicted with diseases such as depression as they reach menopause. In the study of Choi et al. [17], in a similar vein, in the effect of middle-aged women's aerobic dance exercise immersion on psychological well-being, the higher the aerobic immersion, the higher the psychological well-being. Therefore, it is necessary to enhance psychological well-being for a healthier life. Park and Lee reported that middle-aged women are more likely to be depressed because their children grow up and they feel alienated and empty from the sense of separation caused by the increase in their husband's activities outside the home [18].

As women's role burden in work and family life increases, 12% of women are experiencing depression, which is twice that of men [19]. The high prevalence of depression in these women is an important health problem affecting women's quality of life [19]. Depression showed a significant correlation with the quality of life, and low depression showed a high quality of life [20]. As such, the prevalence of depression in women is high, and it is directly related to women's quality of life [21], so it can be said that appropriate nursing intervention is necessary.

Physical, psychological, and social changes in middle-aged women appear in various symptoms. These menopausal symptoms can maintain and promote health in old age, depending on the management, or they can lead to unhealthy conditions, resulting in serious diseases and lowering the quality of life [11]. However, most women do not recognize the symptoms of menopause correctly and think it is a disease, so they spend a lot of time and effort changing hospitals or applying trial and error management methods for symptom relief [21]. Therefore, it is very important and necessary to provide menopause management guidelines that can improve the quality of life of middle-aged women based on the menopausal symptoms and management methods that middle-aged women complain about.

As getting older, the importance of exercise is emphasized [22]. Lack of physical activity leads to hypokinetic diseases such as coronary artery disease, hypertension, diabetes mellitus, obesity, and osteoporosis [22]. Depression is also a big problem, and exercise can help with depression because it stimulates the brain to release endorphins, which makes it feel refreshed after exercise [22]. In menopause, the desire for achievement and concentration decreases, causing psychological loneliness or depression [22]. Physically, as the secretion of hormones decreases, bone density decreases, resulting in osteoporosis and obesity, and the occurrence of cardiovascular diseases increases due to decreased vascular elasticity. It is said that when menopausal women exercise vigorously, muscle tension is relieved and anxiety and nervousness are significantly reduced [22]. Useful exercises for menopausal women include aerobic exercise, weight-bearing exercise, and stretching. Moreover, it is important to maximize compliance in order to continue exercising [23].

## 3. Research Method

### 3.1. Study Design

This study is a cross-sectional quantitative survey study to identify the effects of psychological well-being and depression about menopausal symptoms in middle-aged women using a structured questionnaire.

### 3.2. Respondents of the Study

This study was conducted on middle-aged women (ages 45–60) from group Y in Gangwon-do. Due to the nature of the study, those who underwent hysterectomy and hormone therapy were excluded. Using the G^*∗*^Power 3.1.5 program, the number of samples required for multiple regression analysis was calculated. When the significance level was .05, the power was .95, and the effect size was .15, the calculated sample size was 129. In anticipation of the dropout, 160 copies were distributed, and 155 copies were collected. However, 150 copies were selected, excluding five copies with incomplete or inappropriate responses.

### 3.3. Research Tools

#### 3.3.1. Psychological Well-Being

Psychological well-being refers to feeling joy, meaning, responsibility for life, and achievement of purpose from activities that constitute daily life, having a positive self-image, valuing oneself, and maintaining positive attitudes and emotions [24]. The psychological well-being tool is a tool developed by Yang [25]. The tools used in the study of Park and Kim [26] were employed. This tool is a 14-item, 5-point Likert scale,“ with higher scores indicating higher psychological well-being.” The tool consists of four subfactors: confidence, self-actualization, immersion, and enjoyment. In the study of Yang [25], Cronbach's *α* was .86, whereas, in this study, Cronbach's *α* was .90.

#### 3.3.2. Depression

In this study, the Center for Epidemiology studies of scale (CES-D) developed by Radloff [27] for epidemiologic studies of depression in the general population was used. Park [28] developed a Korean version of the CES-D tool with 20 questions by modifying and supplementing it. This tool consists of seven items of depressive emotion, four items of positive emotion, two items of interpersonal relationship, and seven items of somatic symptoms According to the score, it is classified into four stages:“ not depressed (0–9), slightly depressed (10–15), moderately depressed (16–24), and severely depressed (25 points or higher).” Each item is rated on a Likert scale with “0 points for less than one day, 1 point for one-two days, 2 points for two–four days, and 3 points for five–seven days.” It consists of a minimum of 0 points and a maximum of 60 points. Positive items were inversely converted. A higher score indicates a higher degree of depression. In the study of Park [28], the reliability of the depression tool Cronbach's *α* was 0.92, whereas, in this study, Cronbach's *α* was .94.

### 3.4. Menopausal Symptoms

Menopausal symptoms are symptoms that appear before and after menopause in women, have a comprehensive meaning, and include a series of syndromes caused by endocrine changes related to ovarian function decline, as well as social and psychological factors brought about by changes in the aging process [29]. The menopausal symptom tool was the Menopause Symptom Index (MENSI) developed by Sarrel [30], which was modified and supplemented by Han with 20 items [10]. This tool has 20 items, and each item has “0 points for never, 1 point for sometimes, and 2 points for often,” ranging from 0 to a maximum of 2 points. The higher the score, the higher the menopausal symptoms. The tool consists of three subfactors: physical symptoms, mental symptoms, and sexual symptoms. Cronbach's *α* value was .90 in Han's [16] study, whereas Cronbach's *α* value was .87 in this study.

### 3.5. Ethical Considerations

Respondents who understood the purpose of this study and gave written consent to participate were selected. In order to consider the ethical aspects of the respondents, the purpose of this study and data collection methods were explained, and the subjects were those who voluntarily participated in data collection and gave written consent to participate in the study. They were informed that they could withdraw from participating in the study at any time while the study was in progress. The ethical aspects of the respondents were considered by explaining that the collected data would be anonymous and only used for research purposes and that there would be no exposure of personal information and no disadvantages.

### 3.6. Data Collection Procedure

Data collection was conducted from November 1 to November 30, 2021. The questionnaire was distributed through the local women's center through the research assistant, and the time to fill out the questionnaire was 10 to 15 minutes. The collection rate of the questionnaire was 94%. After signing a written consent form, data were collected using a self-contained questionnaire. The collected personal information is stored on a separate hard disk designated by the researcher and managed independently, and it is not used for any purpose other than the research. The questionnaire used for the research will be stored for 3 years and then incinerated.

### 3.7. Data Analysis Method

The SPSS 21.0 program was used for statistical analysis of the collected data. The differences and levels of psychological well-being, depression, and menopausal symptoms according to demographic and sociological characteristics were analyzed using descriptive statistics, *t*-test, and ANOVA, and the Scheffe's test was used for post hoc testing. The correlation between psychological well-being, depression, and menopausal symptoms was analyzed by Pearson's correlation, and the effect on menopausal symptoms was analyzed by multiple regression.

## 4. Results and Discussion

### 4.1. Difference in Psychological Well-Being, Depression, and Menopausal Symptoms According to General Characteristics

Psychological well-being is first measured by marital status (*F* = 4.45, *P* < 0.05), religion (*t* = 6.30, *P* < 0.05), economic level(*F* = 3.97, *P* < 0.05), regular exercise (*t* = 5.01, *P* < 0.05), hobbies (*t* = 17.40, *P* < 0.001), personality (*t* = 18.66, *P* < 0.001), and subjective health status (*F* = 6.17, *P* < 0.001) and showed a significant difference. Depression was related to marital status (*F* = 4.73, *P* < 0.001), education level (*F* = 2.78, *P* < 0.05), monthly income (*F* = 3.22, *P* < 0.05), living status (*F* = 3.71, *P* < 0.05), regular exercise (*t* = 5.04, *P* < 0.05), hobbies (*t* = 7.79, *P* < 0.05), stress (*t* = 14.48, *P* < 0.001), and personality (*t* = 15.48, *P* < 0.001) and showed a statistically significant difference in their subjective health status (*F* = 5.46, *P* < 0.001). Menopausal symptoms showed significant differences in age (*F* = 3.31, *P* < 0.05), hobbies (*t* = 6.87, *P* < 0.05), and subjective health status (*F* = 7.35, *P* < 0.001) Table 1.

### 4.2. Level of Psychological Well-Being, Depression, and Menopausal Symptoms

The psychological well-being was 46.61 ± 6.92 on a scale of 70 points, and depression was 22.55 ± 9.98 on the scale of 80 points. The score of menopausal symptoms was 8.79 ± 6.43 on the scale of 40, in the subdomain, physical symptoms were 4.06 ± 3.53 on the scale of 18, mental symptoms were 2.72 ± 2.60 on the scale of 14, and sexual symptoms were 2.01 ± 1.71 on the scale of 8 points. The psychological well-being of the subjects was 45.61 ± 6.92 out of 70 points. Depression scored 22.55 ± 9.98 out of a 60-point scale. Menopausal symptoms were 8.79 ± 6.43 out of 40 points, physical symptoms were 4.06 ± 3.53 out of 18 points, mental symptoms were 2.72 ± 2.60 out of 14 points, and sexual symptoms were 2.01 ± 1.71 out of 8 points Table 2.

### 4.3. Correlation between Psychological Well-Being, Depression, and Menopausal Symptoms

The subject's psychological well-being was characterized by depression (*r* = −0.431, *P* < 0.001), menopausal symptoms (*r* = −0.358, *P* < 0.001), physical symptoms (*r* = −0.344, *P* < 0.001), and mental symptoms (*r* = −0.352, *P* < 0.001) and was found to have a significant negative correlation. Depression was characterized by menopausal symptoms (*r* = 485, *P* < 0.001), physical symptoms (*r* = 410, *P* < 0.001), psychological symptoms (*r* = 492, *P* < 0.001), and sexual symptoms (*r* = 228, *P* < 0.001) and was found to have a significant positive correlation. Menopausal symptoms showed a significant positive correlation between physical symptoms (*r* = 893, *P* < 0.001), mental symptoms (*r* = 861, *P* < 0.001), and sexual symptoms (*r* = 609, *P* < 0.001) (Table 3).

### 4.4. Factors Affecting Menopausal Symptoms

Prior to the regression analysis, whether multicollinearity occurred between each variable was checked. The tolerance limit values ranged from 0.80 to 0.81, which were all greater than 0.1, and the dispersion expansion values were 1.055 to 1.282, all not exceeding 10, indicating that there was no problem with multicollinearity. Statistically significant variables include depression and psychological well-being in multiple regression analysis. The factors affecting menopausal symptoms were statistically significant in the order of depression (*β* = .405, *P* < 0.001) and psychological well-being (*β* = −0.184, *P* < 0.05). Psychological well-being was analyzed to have the opposite effect on menopausal symptoms, and the factors used in the analysis had an explanatory power of menopausal symptoms 25.2% Table 4.

Exercise that showed a statistically significant difference can be viewed as an important, actionable intervention that can alleviate menopausal symptoms through individual habit change. The effect of maintaining health through exercise improves overall physical strength such as positive changes in blood lipid components, stabilization of the endocrine system, increase in lung capacity, strengthening of muscle strength, and weight loss [31]. In addition, it plays an important role in health management, such as preventing chronic diseases (e.g., cardiopulmonary disease, lipid metabolic disease, osteoporosis, and obesity) and improving health status [31]. In particular, it explains that regular or active exercise during menopause is an effective way to cope with the physical and mental changes frequently observed in menopause [31]. Increased secretion of hormones such as endorphin, estriol, and testosterone due to exercise relieves negative emotions such as anxiety, depression, and stress and increases sexual libido [32]. In addition, by continuously maintaining social friendships and social activities, they have positive thoughts and stable emotional states. Therefore, exercise intervention for menopausal women is considered a good way to relieve menopausal symptoms and maintain and promote the overall health of menopausal women [33].

The depression score of this study was 37.57 (100 points converted). In the study of Yang [25] using the same measurement tool, the depression score was 35.93 (100 points converted), which is similar to this study. In the study of Kim [19], the depression score was 22.38 points (100 points converted), which was lower than that of this study. The subjects of this study were ordinary middle-aged women without any affiliation, but Kim's subjects were middle-aged women who attend Church [19]. It is thought that middle-aged women who belonged to a Church group had more emotional stability due to a sense of belonging to the group.

The average menopausal symptoms of the study subjects were 8.79 points. This study's score of 8.79 was lower than the Kim Ji-young study's score of 10.09 for menopausal symptoms [19] and 15.16 points in the Kim et al.'s study [12]. Because there were relatively more subjects who had menopause than in this study, it seems that the scores for menopausal symptoms were rather high. Sexual symptoms were the most common among menopausal symptoms in this study. Based on Kim Ji-young's study, physical symptoms were the highest among menopausal symptoms [15], and Han Sook-hee's study reported the highest psychological symptoms [16], whereas, in Kim Su-jin's study, sexual symptoms were reported the most, which was consistent with this study [31]. As such, middle-aged women are complaining of various symptoms in all areas,of mental and sexual as well as physical symptoms. Therefore, it is considered that a follow-up study is necessary because there are various differences depending on the study.

Multiple regression analysis of middle-aged women's psychological well-being and depression yielded statistically significant findings with depression and psychological well-being as variables influencing menopausal symptoms. In particular, psychological well-being was found to have a negative effect on menopausal symptoms, which means that the higher the psychological well-being, the lower the menopausal symptoms. It demonstrates that making participants experience psychological and emotional well-being is a key role in relieving menopausal symptoms in middle-aged women.

In order to reduce menopausal symptoms in middle-aged women who play an important part in the developmental stage to lead to a happy old age, various interventions are needed to improve psychological well-being and reduce depression. In addition, among the factors that showed significant results for menopausal symptoms, exercise and hobbies, which were shown to be factors that can alleviate menopausal symptoms due to individual lifestyle changes, are encouraged, which will contribute to reducing menopausal symptoms and improving the quality of life.

## 5. Conclusions

The purpose of this study was to provide basic data on the health by examining the effects of psychological well-being and depression on menopausal symptoms and the necessity of exercise in middle-aged women.

Psychological well-being showed significant differences in marital status, religion, economic level, regular exercise, hobbies, personality, and subjective health status. Depression showed significant results in marital status, education level, monthly income, cohabitation, regular exercise, hobbies, stress, personality, and subjective health status. Menopausal symptoms showed significant results in age, regular exercise, hobbies, and subjective health status. Depression showed a positive correlation with menopausal symptoms, whereas psychological well-being showed a negative correlation with depression and menopausal symptoms. In addition, it was found that menopausal symptoms had an effect on depression and psychological well-being in the order.

In order to reduce menopausal symptoms in middle-aged women, various interventions are needed to improve psychological well-being and reduce depression. In addition, it is expected that it will contribute to reducing menopausal symptoms and improving quality of life by recommending exercise activities that have been shown to be a factor that can alleviate menopausal symptoms through individual lifestyle changes among the factors that showed significant results for menopausal symptoms.

The following suggestions are made: First, since there are not enough previous studies targeting middle-aged women, many follow-up studies with various variables should be conducted. Second, although it was aimed at middle-aged women, many studies on middle-aged men should be conducted in the future. Third, although the questionnaire method was used in this study, it is considered that many qualitative research methods should be conducted in subsequent studies.

## Figures and Tables

**Table 1:** Difference in psychological well-being, depression, and menopausal symptoms according to general characteristics (*N* = 150).

Characteristics	Categories		*n* (%)	Psychological well-being		Depression		Menopausal symptoms	
				*M* ± SD	*T*/*F*(*p*) Scheffe	*M* ± SD	*T*/*F*(*p*) Scheffe	*M* ± SD	*T*/*F*(*p*), Scheffe
Age (year) 48.76 ± 6.18	45∼49	*a*	85 56.7)	46.96 ± 7.29	0.35 (0.705)	22.63 ± 9.96	1.11 (0.330)	7.63 ± 5.94	3.32 (0.039)*b*, *c* > *a*
	50∼59	*b*	57 (38)	46.29 ± 6.27		21.98 ± 9.51		10.40 ± 6.74	
	≧60	*c*	8 (5.3)	45.12 ± 7.77		26.15 ± 1.10		9.62 ± 7.52	

Marital status	Unmarried	*a*	18 (12)	42.33 ± 7.03	4.45 (0.002), *d*, *b*, *c*, *a* > e	26.29 ± 13.75	4.73 (0.001), *d*, e, *a*, *c* > *b*	10.66 ± 6.95	1.59 (0.178)
	Married	*b*	119 (79.3)	47.57 ± 6.48		21.36 ± 8.31		8.14 ± 6.30	
	Death of a spouse	*c*	5 (3.3)	47.40 ± 6.34		25.50 ± 12.76		12.00 ± 7.51	
	Separation	*d*	2 (1.3)	48.00 ± 1.41		34.13 ± 10.60		12.00 ± 5.65	
	Divorce	*e*	6 (4.0)	39.16 ± 8.79		28.50 ± 11.67		12.33 ± 5.46	

Education	Primary school	*a*	2 (1.3)	42.00 ± 5.65	1.00 (0.409)	32.63 ± 19.09	2.78 (0.029), *a*, *b*, *c*, *d* > e	18.50 ± 10.60	1.391 (0.240)
	Middle school	*b*	3 (2.0)	44.00 ± 4.35		30.50 ± 10.78		11.33 ± 12.34	
	High school	*c*	21 (14)	4.604 ± 7.25		23.71 ± 8.10		9.38 ± 6.79	
	University	*d*	93 (62)	46.29 ± 7.10		22.57 ± 10.21		8.43 ± 6.06	
	Graduate school	*e*	31 (20.7)	48.51 ± 6.26		20.27 ± 8.05		8.61 ± 6.40	
	No		59 (39.3)	44.88 ± 7.09		23.68 ± 10.83		9.83 ± 6.29	

Occupation	Housewives		19 (12.7)	47.47 ± 6.30	1.35 (0.236)	23.60 ± 8.80	1.09 (0.370)	7.00 ± 7.45	1.08 (0.374)
	Civil servant		36 (24)	46.41 ± 6.76		20.96 ± 7.73		8.22 ± 5.45	
	Professional/Management		39 (26)	48.20 ± 6.69		21.26 ± 8.76		9.69 ± 6.79	
	Office		25 (16.7)	45.00 ± 6.20		23.25 ± 11.16		9.32 ± 6.91	
	Sales service		3 (2)	38.66 ± 10.59		25.50 ± 13.74		6.66 ± 2.51	
	Self-employment		3 (2)	44.33 ± 7.96		26.50 ± 19.08		15.66 ± 11.06	
	Other		25 (16)	46.60 ± 7.96		24.51 ± 11.81		8.48 ± 5.42	

Month income (10,000 won)	≥100	*a*	2 (1.3)	39.50 ± 2.12	2.09 (0.085)	32.25 ± 14.14	3.22 (0.014) e > *d*, *c*, *b* > *a*	18.50 ± 9.19	1.87 (0.119)
	100∼200	*b*	16 (10.7)	46.93 ± 7.44		25.50 ± 10.32		9.18 ± 7.39	
	200∼300	*c*	38 (25.3)	44.36 ± 7.50		24.41 ± 10.74		9.57 ± 6.16	
	300∼400	*d*	37 (24.7)	47.51 ± 6.97		21.41 ± 8.40		7.24 ± 6.57	
	400≤	*e*	57 (38)	47.68 ± 6.09		20.88 ± 9.15		8.82 ± 5.98	

Living status	Alone	*a*	17 (11.3)	44.52 ± 8.89	1.33 (0.266)	26.60 ± 2.81	3.71 (0.027) *a* > *b* > *c*	10.35 ± 7.21	1.41 (0.250)
	Family	*b*	130 (86.7)	46.97 ± 6.66		22.15 ± 9.28		8.48 ± 6.35	
	Friends or colleagues	*c*	3 (2)	50.66 ± 2.88		17.00 ± 4.61		13.33 ± 3.21	

Economic state	Abundance	*a*	8 (5.3)	51.62 ± 10.64	3.97 (0.021) *a* > *b* > *c*	23.90 ± 3.56	1.51 (0.223)	7.37 ± 5.90	2.22 (0.112)
	No difficulty	*b*	117 (78)	46.81 ± 6.19		22.00 ± 9.66		8.37 ± 6.23	
	Difficulty	*c*	25 (16.7)	44.08 ± 7.98		24.69 ± 9.31		11.20 ± 7.21	

Regular exercise	Yes		52 (34.7)	48.32 ± 6.47	5.01 (0.027)	20.71 ± 8.72	5.04 (0.026)	7.17 ± 5.92	5.18 (0.024)
	No		98 (65.3)	45.70 ± 7.00		23.52 ± 10.22		9.65 ± 6.56	

Hobby	Yes		46 (30.7)	49.97 ± 6.16	17.40 (0.000)	20.07 ± 7.92	7.79 (0.006)	6.76 ± 5.45	6.87 (0.010)
	No		104 (69.3)	45.12 ± 6.73		23.64 ± 10.30		9.69 ± 6.65	

Stress situation (in the past year)	Yes		38 (25.3)	47.23 ± 6.98	0.41 (0.522)	26.33 ± 9.42	14.48 (0.000)	10.39 ± 7.46	3.19 (0.076)
	No		112 (74.7)	46.40 ± 6.91		21.26 ± 9.45		8.25 ± 5.99	

Personality	Positive		128 (85.3)	47.57 ± 6.74	18.66 (0.000)	21.61 ± 8.88	15.48 (0.000)	8.48 ± 6.03	2.02 (0.157)
	Negative		22 (14.7)	41.04 ± 5.13		28.02 ± 12.14		10.59 ± 8.38	

Subjective health state	Very healthy	*a*	3 (2)	55.33 ± 5.13	6.17 (0.000) *a* > *b*, *c*, e > *d*	18.25 ± 3.21	5.46 (0.000) e > *d* > *c*, *b*, *a*	5.33 ± 5.77	7.35 (0.000) e > *d*, *c* > *b*, *a*
	General health	*b*	67 (44.7)	48.82 ± 6.48		20.62 ± 7.65		6.32 ± 4.76	
	Usually	*c*	62 (41.3)	45.04 ± 6.59		23.36 ± 10.86		10.43 ± 6.74	
	Slight disease	*d*	16 (10.7)	42.18 ± 5.79		26.34 ± 10.03		11.93 ± 6.89	
	Serious disease	*e*	2 (1.3)	43.50 ± 10.60		38.25 ± 1.41		20.50 ± 9.19	

**Table 2:** Score of psychological well-being, depression, and menopausal symptoms (*N* = 150).

Variable	Range	M ± SD
Psychological well-being	14 ∼ 70	46.61 ± 6.92
Depression	0 ∼ 60	22.55 ± 9.86
Menopausal symptoms	0 ∼ 40	8.79 ± 6.43
Physical symptoms	0∼18	4.06 ± 3.53
Mental symptoms	0∼14	2.72 ± 2.60
Sexual symptoms	0∼8	2.01 ± 1.71

**Table 3:** Correlation between psychological well-being, depression, and menopausal symptoms (*N* = 150).

Variable	Psychological well-being	Depression	Menopausal symptoms	Subscales		
				Physical symptoms	Mental symptoms	Sexual symptoms
Psychological well-being	1					
Depression	−0.431^*∗∗*^	1				
Menopausal symptoms	−0.358^*∗∗*^	0.485^*∗∗*^	1			
Physical symptoms	−0.344^*∗∗*^	0.410^*∗∗*^	0.893^*∗∗*^	1		
Mental symptoms	−0.352^*∗∗*^	0.492^*∗∗*^	0.861^*∗∗*^	0.637^*∗∗*^	1	
Sexual symptoms	−0.102	0.228^*∗∗*^	0.609^*∗∗*^	0.328^*∗∗*^	0.404^*∗∗*^	1

^*∗*^ *P* < 0.05, ^*∗∗*^*P* < 0.001.

**Table 4:** Factors affecting menopausal symptoms.

Variable	B	SE	*β*	t	*P*
(Constant)	8.793	4.324		2.034	<0.05
Psychological well-being	−0.171	0.073	−0.184	−2.338	<0.05
Depression	0.265	0.051	0.405	5.165	<0.001
	Adj *R*^2^ = 0.252	*R * ^2^ = 0.262	*F* = 25.12	*P* < 0.001	

## Data Availability

This data presented in this study are available on the electronic journal website.
